# Flutamide-Induced Cytotoxicity and Oxidative Stress in an *In Vitro* Rat Hepatocyte System

**DOI:** 10.1155/2014/398285

**Published:** 2014-10-13

**Authors:** Abdullah Al Maruf, Peter O'Brien

**Affiliations:** ^1^Department of Pharmacology & Toxicology, Faculty of Medicine, University of Toronto, Toronto, ON, Canada M5S 1A8; ^2^Leslie Dan Faculty of Pharmacy, University of Toronto, Toronto, ON, Canada M5S 3M2

## Abstract

Flutamide (FLU) is a competitive antagonist of the androgen receptor which has been reported to induce severe liver injury in some patients. Several experimental models suggested that an episode of inflammation during drug treatment predisposes animals to tissue injury. The molecular cytotoxic mechanisms of FLU in isolated rat hepatocytes using an *in vitro* oxidative stress inflammation system were investigated in this study. When a nontoxic hydrogen peroxide (H_2_O_2_) generating system (glucose/glucose oxidase) with peroxidase or iron(II) [Fe(II)] (to partly simulate *in vivo* inflammation) was added to the hepatocytes prior to the addition of FLU, increases in FLU-induced cytotoxicity and lipid peroxidation (LPO) were observed that were decreased by 6-*N*-propyl-2-thiouracil or deferoxamine, respectively. *N*-Acetylcysteine decreased FLU-induced cytotoxicity in this system. Potent antioxidants, for example, Trolox ((±)-6-hydroxy-2,5,7,8-tetramethylchroman-2-carboxylic acid), resveratrol (3,5,4′-trihydroxy-*trans*-stilbene), and DPPD (*N,N*′-diphenyl-1,4-phenylenediamine) also significantly decreased FLU-induced cytotoxicity and LPO and increased mitochondrial membrane potential (MMP) and glutathione (GSH) levels in the H_2_O_2_ generating system with peroxidase. TEMPOL (4-hydroxy-2,2,6,6-tetramethylpiperidin-1-oxyl), a known reactive oxygen species (ROS) scavenger and superoxide dismutase mimetic, also significantly decreased toxicity caused by FLU in this system. These results raise the possibility that the presence or absence of inflammation may be another susceptibility factor for drug-induced hepatotoxicity.

## 1. Introduction

Flutamide (FLU) is a competitive antagonist of the androgen receptor, which is used, in association with castration, in the treatment of metastatic prostatic carcinoma [1]. The efficacy of this antiandrogen is somewhat overshadowed by the occurrence of hepatitis in a few subjects. The incidence of hepatotoxicity (defined as >4-fold increase in serum transaminase activity) has been found to be 0.36% of 1091 consecutively treated patients with prostate cancer [2].

Unlike other nitroaromatic drugs, FLU (chemical structure is presented in Figure 1) was not noticeably reduced into a nitroanion free radical by NADPH- (nicotinamide adenine dinucleotide phosphate-) cytochrome P450 reductase. Instead, rat and human microsomal cytochrome P450 oxidatively metabolized FLU into electrophilic metabolite(s), which bound covalently to microsomal proteins [3]. FLU is metabolized into 2-hydroxy FLU in liver by the CYP1A2. FLU is also known to be metabolized into 4-nitro-3(trifluoromethyl)phenylamine [4]. FLU and 2-hydroxy FLU were cytotoxic to primary cultured rat hepatocytes at concentrations of approximately 40 *µ*M and 170 *µ*M, respectively [5]. FLU (1 mM) decreased the reduced glutathione/glutathione disulfide (GSH/GSSG) ratio and total protein thiols. The addition of cystine (a GSH precursor) increased GSH and decreased lactate dehydrogenase (LDH) release in male rat hepatocytes [6]. FLU (50 *µ*M) markedly inhibited complex I respiration in isolated male rat liver mitochondria and FLU (1 mM) also decreased adenosine 5′-triphosphate (ATP) levels in isolated male rat hepatocytes [6]. Fau and colleagues [6] suggested that FLU is toxic to rat hepatocytes as a result of cytochrome P450- (3A- and 1A-) mediated electrophilic metabolite(s) formation, whose damaging effects are aggravated by the inhibitory effect of FLU on mitochondrial respiration and ATP formation.

Some FLU-induced liver cases were found to be associated with blood eosinophilia and neutropenia, suggesting the involvement of the immune system [7, 8]. It was suggested that, in some individuals, FLU may render hepatocytes more susceptible to oxidant-mediated injury that can initiate infiltration of polymorphonuclear neutrophils (PMNs) in the liver and increase PMN responsiveness to endogenous activators [9].

Inflammation is a necessary response to pathogen invasion. However, inappropriate or unregulated inflammatory reactions may cause tissue injury. Before drug-induced liver injury occurs* in vivo*, an inflammatory response usually occurs and cells other than hepatocytes (e.g., Kupffer cells, macrophages) become activated. Inflammation caused by infections or endotoxin markedly activates NADPH oxidase thereby forming hydrogen peroxide (H_2_O_2_) [10, 11]. NADPH oxidases are membrane-bound enzyme complexes found in the membranes of phagosomes and are used by neutrophils and white blood cells to engulf microorganisms. Normally, the complex, Gp91PHOX (contains heme) (encoded by gene* Nox2*), is latent in neutrophils and is activated during the respiratory burst [10]. They have been implicated as a major source of ROS generation [12]. When a phagocytic cell is exposed to invading foreign compounds or their degradation products or metabolites, the defense enzyme (NADPH oxidase) undergoes a series of reactions called the “respiratory burst” that enable the cell to provide oxidizing agents (ROS) to destroy such compounds [13]. When NADPH oxidase becomes activated, it catalyzes the NADPH-dependent reduction of oxygen to superoxide (O_2_^•−^) within the plasma membrane or on its outer surface (Figure 2). Another strong oxidant and antimicrobial agent, hypochlorous acid (HOCl), can also be formed from H_2_O_2_ catalyzed by myeloperoxidase (MPO) (Figure 2). Immune cells (e.g., neutrophils and macrophages) also infiltrate the liver [13, 14]. It has been suggested that the H_2_O_2_ and MPO from the infiltrated cells catalyze the oxidation of drugs (or their metabolites) to form reactive prooxidant radicals that are toxic to hepatocytes (Scheme 1) [10, 15]. Numerous studies with animals have shown that a modest inflammatory response enhances tissue susceptibility to drugs/xenobiotics (reviewed in [11]).

In order to simulate the marked increase of drug-induced hepatotoxicity caused by acute episodes of inflammation* in vivo,* our laboratory has developed an* in vitro *hepatocyte screening system which includes subjecting freshly isolated rat hepatocytes to a nontoxic continuous flow of a H_2_O_2_ generating system using glucose (G) and glucose oxidase (GO) and supplementing it with either horseradish peroxidase (HRP) or Fe(II) to partly simulate* in vivo *inflammation. We also test what compounds or antioxidants may act as antidotes to prevent or delay drug-induced cytotoxicity using accelerated cytotoxicity mechanism screening (ACMS) techniques [16] (Scheme 1) in freshly isolated rat hepatocytes.

Early in drug discovery,* in vitro* cytotoxicity is becoming increasingly recognized as an effective indicator of human toxicity potential that must be addressed in order to maximize probability of successful progression of compounds into development. The ACMS methods determine the molecular cytotoxic mechanisms of drugs/xenobiotics when incubated at 37°C for 3 hrs using freshly isolated rat hepatocytes. This functionomic approach is useful for understanding the molecular cytotoxic mechanisms of drugs/xenobiotics under investigation. A major assumption with ACMS is that high dose/short duration (*in vitro*) exposure simulates low dose/long duration (*in vivo*) exposure [16]. Our laboratory successfully uses ACMS techniques to investigate molecular mechanisms of drug/xenobiotic-induced cytotoxicity in isolated rat hepatocytes. Recent examples include azathioprine [17], chlorpromazine [18], hydralazine [19], amodiaquine [20], and polychlorinated biphenyls [21].

Previously we showed that FLU-induced cytotoxicity can be increased in the presence of H_2_O_2_ and HRP [10]. In this study, we further investigated FLU-induced cytotoxicity mechanisms by adding Fe(II) to the system and determining compounds that can prevent or decrease FLU-induced hepatotoxicity in the presence of an* in vitro* oxidative stress inflammation system. We hypothesize that exposure of FLU to the* in vitro* oxidative stress inflammation system will increase hepatotoxicity through the formation of prooxidant radicals and other ROS leading to oxidative stress. A simplified schematic representation of the hypothesis and aims of the study is presented in Scheme 1.

## 2. Materials and Methods

### 2.1. Chemicals

Flutamide (2-methyl-*N*-[4-nitro-3-(trifluoromethyl)phenyl]-propanamide), glucose oxidase from* Aspergillus niger* (type II, 15,000–50,000 units/g solid), peroxidase from horseradish (type II, 150–250 units/mg solid), 6-*N*-propyl-2-thiouracil (PTU),* N*-acetyl-*L*-cysteine (NAC), (±)-6-hydroxy-2,5,7,8-tetramethylchroman-2-carboxylic acid (Trolox), 4-hydroxy-2,2,6,6-tetramethylpiperidin-1-oxyl (TEMPOL),* N*,*N*′-diphenyl-*p*-phenylenediamine (DPPD), resveratrol (3,5,4′-trihydroxy-*trans*-stilbene), and all other chemicals were purchased from Sigma-Aldrich Corp. (Oakville, ON, Canada). Type II collagenase (from* Clostridium histolyticum*) was purchased from Worthington Biochemical Corp. (Lakewood, NJ, USA). 4-(2-Hydroxyethyl) piperazine-1-ethanesulfonic acid (HEPES) was purchased from Boehringer-Mannheim Ltd. (Montreal, QC, Canada).

### 2.2. Animals

Male Sprague-Dawley rats (Charles River Laboratories International Inc., Wilmington, MA, USA) weighing 275–300 g were used for experimental purposes. Experiments were carried out in compliance with the* Guide to the Care and Use of Experimental Animals by Canadian Council on Animal Care* [22]. The University of Toronto Animal Use Protocol was reviewed and approved by the Faculty of Medicine and Pharmacy Animal Care Committee. Rats were housed in ventilated plastic cages with 12 air changes per hr, 12 hr light photoperiod (lights on at 08:00), and an environmental temperature of 21–23°C with 50–60% relative humidity. The animals were fed a normal standard chow diet and water* ad libitum*.

### 2.3. Hepatocyte Preparation

Hepatocytes were isolated from rats using collagenase perfusion of the liver [23]. Isolated hepatocytes (10 mL, 10^6^ cells/mL) were suspended in Krebs-Henseleit buffer (pH 7.4) containing 12.5 mM HEPES in continually rotating 50 mL round bottom flasks, under an atmospheric condition of 95% O_2_ and 5% CO_2_ in a 37°C water bath for 30 min prior to the addition of chemicals.

### 2.4. *In Vitro* Oxidative Stress Inflammation System

A H_2_O_2_ generating system was employed by adding 10 mM G to the hepatocyte suspension followed by GO (0.5 unit/mL). This G/GO system continuously supplied H_2_O_2_ during the 3 hr experimental period, without affecting GSH levels or cell viability. FLU was coincubated with the H_2_O_2_ generating system and HRP (0.5 *μ*M). HRP was preincubated with hepatocytes for 15 min prior to the addition of other agents. Peroxidase activity was inhibited by PTU (5 *μ*M) [24] by preincubating it with hepatocytes for 15 min prior to the start of the experiment. FLU was also incubated with the Fe(II)-mediated Fenton model, which consisted of nontoxic concentrations of Fe(II) [2 *μ*M Fe(II) and 4 *μ*M 8-hydroxyquinoline (8-HQ)] with the H_2_O_2_ generating system [10]. Deferoxamine (200 *μ*M) was added to chelate Fe(II) and was preincubated with hepatocytes for 30 min prior to the addition of other agents. The concentrations of H_2_O_2_ generating system/antioxidants/ROS-scavengers/Fenton system/Fe(II)-chelator used in the experiments had no significant effect on hepatocyte viability at the concentrations used.

### 2.5. Cell Viability

Hepatocyte viability was assessed by the trypan blue (0.1% w/v) exclusion assay [23]. Hepatocyte viability was determined at every 60 min during a 3-hour incubation period. Only cell preparations with viability of 80–90% were used for the experiments.

### 2.6. Reactive Oxygen Species Formation (ROS) Assay

Hepatocyte ROS generation was determined using 2′,7′-dichlorofluorescein diacetate (DCFD) which can permeate hepatocytes and be deacetylated by intracellular esterases to form nonfluorescent dichlorofluorescin (DCF). DCF is oxidized by intracellular ROS to form the highly fluorescent dichlorofluorescein. ROS formation was assayed by withdrawing 1 mL hepatocyte samples at 30 and 90 mins, which were then centrifuged for 1 min at 5000 ×g. The cells were resuspended in Krebs-Henseleit buffer and 1.6 *μ*M DCFD was added. The cells were incubated at 37°C for 10 min, and the fluorescent intensity of dichlorofluorescein was measured using a SPECTRAmax Gemini XS spectrofluorometer (Molecular Devices, Sunnyvale, CA, USA) set at 490 nm excitation and 520 nm emission wavelengths [25] and was expressed as FI (fluorescence intensity) unit.

### 2.7. Lipid Peroxidation (LPO) Assay

LPO was determined by measuring the amount of thiobarbituric acid reactive substances (TBARS) formed during the decomposition of lipid hydroperoxides, mostly formed from malondialdehyde (MDA) with the pink adduct being measured at 532 nm. Each test tube containing 1 mL aliquots of hepatocyte suspension (withdrawn at 30 and 90 mins) was treated with 250 *μ*L of trichloroacetic acid (70% w/v) and 1 mL of thiobarbituric acid (0.8% w/v). The suspension was then boiled for 20 min in a boiling water bath. The samples were cooled for 5 min and then centrifuged at 5000 ×g for 5 min. The supernatant was measured at 532 nm to detect the amount of TBARS formed during the decomposition of lipid hydroperoxides, using a SPECTRAmax Plus 384 spectrophotometer (Molecular Devices, Sunnyvale, CA, USA). Results were expressed as *µ*M concentration of MDA (156 mM^−1^ cm^−1^) [26].

### 2.8. Glutathione (GSH) Assay

GSH in hepatocytes was determined colorimetrically at 412 nm at 30 and 90 mins by commercial kits from Cayman Chemical, Ann Arbor, MI, USA, according to the manufacturer's instruction. GSH values were calculated according to Bulteau and colleagues [27] and were expressed as nmoles/10^6^ cells.

### 2.9. Mitochondrial Membrane Potential (MMP) Assay

MMP was estimated by measuring the uptake of the cationic fluorescent dye, rhodamine 123, into hepatocytes. Aliquots (500 *μ*L) of the cell suspension were separated at 30 and 90 mins from the incubation medium by centrifugation at 5000 ×g for 1 min. The cell pellet was resuspended in 2 mL of fresh incubation medium containing 1.5 *μ*M rhodamine 123 and incubated at 37°C in a thermostatic water bath for 10 min with gentle shaking. Hepatocytes were then separated by centrifugation and the amount of rhodamine 123 remaining in the incubation medium was measured at 490 nm excitation and 520 nm emission wavelengths using a SPECTRAmax Gemini XS spectrofluorometer (Molecular Devices, Sunnyvale, CA, USA). The capacity of mitochondria to take up the rhodamine 123 dye was calculated as the difference in fluorescence intensity between control and treated cells and was expressed as % MMP compared to control hepatocytes [28].

### 2.10. Statistical Analysis

The SPSS software package (version 14.0, SPSS Inc., Chicago, IL, USA) was used to analyze the data. Values were rounded and were expressed as mean ± standard error of the mean (SEM) from 3 independent experiments. Statistical analysis was performed using one-way analysis of variance (ANOVA) and Tukey's post hoc test to assess significance between control and treatment groups in these experiments. *P* < 0.05 was considered significant.

## 3. Results 

A concentration- and time-dependent increase in cytotoxicity (Figure 3), ROS formation, and a decrease in % MMP (data not shown) were observed for FLU (50–100 *µ*M) compared to control hepatocytes over 3 hours of the incubation period. Incubation of freshly isolated rat hepatocytes for 2 hrs at 37°C with 75 *µ*M FLU induced an approximate 50% loss in hepatocyte viability as measured by the trypan blue exclusion assay (LC_50_, according to the ACMS techniques). We used the LC_50_ value (lethal concentration required to cause 50% cytotoxicity in 2 hrs at 37°C) to investigate potential cytotoxic mechanisms of the drug or xenobiotic under investigation [16].

In a previous study, the addition of a nontoxic H_2_O_2_ generating system with HRP (0.5 *µ*M) caused a significant increase in FLU- (75 *µ*M) induced cytotoxicity [10]. This was significantly decreased by the addition of PTU (5 *µ*M) (a peroxidase inhibitor) (Figure 4) in the current study. Furthermore, with the addition of a H_2_O_2_ generating system and HRP, a significant increase in LPO (MDA equivalents, *µ*M) and a decrease in % MMP (Table 1) and GSH levels (Figure 5) compared to control hepatocytes were noted. Similar results were obtained when we used the Fenton model (a nontoxic H_2_O_2_ generating system and Fe(II) that generates hydroxyl radicals). An iron chelator, deferoxamine (200 *µ*M, preincubated for 30 min), decreased FLU-induced cytotoxicity likely by inhibiting the Fenton reaction (Figure 4).

A significant decrease in GSH levels was observed when FLU was administered with the H_2_O_2_ generating system and peroxidase to isolated rat hepatocytes (Figure 5). This was prevented by 1 mM* N*-acetylcysteine (a GSH precursor) (Figure 5). Potent antioxidants, Trolox (1 mM), resveratrol (50 *µ*M), and DPPD (2 *µ*M) also significantly decreased FLU-induced cytotoxicity and LPO and increased % MMP (Table 1) and GSH levels (Figure 5) in this system compared to control hepatocytes. Significant protection against FLU-induced cytotoxicity with the H_2_O_2_ generating system and peroxidase was also achieved by a ROS scavenger, TEMPOL (200 *µ*M) (Table 1). All modulating agents were noncytotoxic compared to control hepatocytes at the concentrations used.

## 4. Discussion

Inflammatory episodes are common in people and animals and are precipitated by numerous stimuli such as bacteria, viruses, and exposure to toxins produced by microorganisms. Inflammagens such as lipopolysaccharide can also activate Kupffer cells (resident liver macrophages) and other inflammatory cells in the liver (reviewed in [11]). Immune cells (e.g., neutrophils and macrophages) also infiltrate the liver. Inflammation caused by infections or endotoxins markedly activates NADPH oxidase thereby forming H_2_O_2_. Whilst there is little peroxidase activity in hepatocytes, MPO is located in Kupffer cells of the human and rodent liver [29]. Neutrophil infiltration of the liver in response to inflammation can result in a 50- to 100-fold increase in hepatic MPO activity [30]. Peroxidase and H_2_O_2_ can also oxidatively activate/detoxify some drugs/xenobiotics at a higher peroxidase dose (Scheme 1) [10, 15].

Several experimental models have suggested that an episode of inflammation during drug treatment predisposes the animals to tissue injury and may be an important determinant of individual susceptibility to the drug (reviewed in [11]). Therefore, it is important to define the role of inflammation in drug toxicity and to develop models or methods to predict which drugs or drug candidates have the potential to cause toxicity through interaction with inflammation. This knowledge could allow identification of individuals who are susceptible to inflammation-enhanced toxicity and a better understanding of the confluence of events required for this type of adverse response [10, 11, 15].

The “*In Vitro* Oxidative Stress Inflammation System” involves subjecting freshly isolated rat hepatocytes to a low, noncytotoxic continuous flow of H_2_O_2_ (using G and GO) and supplementing it with either HRP or Fe(II) to partly simulate* in vivo *inflammation (Scheme 1). HRP/H_2_O_2_ was used for* in situ* activation of drugs and for simulating MPO. The H_2_O_2_ acts by increasing the oxidation state of the ferric iron which then oxidizes the peroxidase substrates (reviewed in [31]). PTU was used as a peroxidase inhibitor in this study as evidence for the involvement of HRP/H_2_O_2_-catalyzed formation of prooxidant radicals from drug and/or its metabolites. PTU inhibits HRP in a noncompetitive form [32]. Phagocytes generate O_2_^•−^ radicals and H_2_O_2_ and their interaction results in Fe(II)-catalyzed reaction that forms hydroxyl radical (^•^OH) (Scheme 1). Deferoxamine chelates Fe(II) in a catalytically inactive form, and thus inhibition by deferoxamine has been employed as evidence for the involvement of ^•^OH generated by the Fenton reaction [33]. Although use of high concentrations of the drug is a limitation of this* in vitro* study, ACMS techniques assume that the drug metabolic/toxic pathways at cytotoxic drug concentrations* in vitro* at 2 hrs are similar to those that occur* in vivo* at 24–36 hrs [16]. With 24 halobenzenes, it was found that the relative lethal concentrations required to cause 50% cytotoxicity in 2 hrs at 37°C (defined as ACMS LC_50_), as determined* in vitro* using hepatocytes isolated from phenobarbital-induced Sprague-Dawley rats, correlated with hepatotoxicity* in vivo* at 24–54 hrs [34]. Moreover, using these techniques, the molecular hepatocytotoxic mechanisms found* in vitro* for six classes of xenobiotics/drugs were found to be similar to the rat hepatotoxic mechanisms reported* in vivo* [35]. However, the mechanism of toxicity at higher drug concentrations than clinical drug concentrations is not always the same as at clinically relevant drug concentrations. Caution should be taken in interpretation of the results in humans.

Addition of a nontoxic H_2_O_2_ generating system with HRP caused a significant increase in FLU-induced cytotoxicity and LPO and a decrease in % MMP (Table 1) and GSH levels (Figure 5) that was significantly decreased by the addition of PTU (a peroxidase inhibitor) (Figure 4). Similar results were obtained when we used the Fenton model. An iron chelator, deferoxamine, was found to decrease FLU-induced cytotoxicity (Figure 4). This suggests that using the Fenton system to generate ^•^OH increased hepatocyte susceptibility to FLU-induced cytotoxicity, almost similar to that of the nontoxic H_2_O_2_ and HRP system. Srinivasan and colleagues [9] suggested that in some individuals FLU simultaneously renders hepatocytes more susceptible to oxidant-mediated injury that can initiate infiltration of PMNs into the liver and increases PMN responsiveness to endogenous activators. The incidence of FLU-induced hepatotoxicity was found in only 0.36% of 1091 consecutively treated patients with prostate cancer indicating that most patients do not experience liver toxicity. Furthermore, FLU-induced hepatotoxicity is often associated with inflammation [2, 36]. Some cases were found to be associated with blood eosinophilia [7]. Therefore, it can be speculated that an episode of inflammation during FLU therapy could decrease the threshold for FLU toxicity and thereby render an individual susceptible to a toxic reaction that would otherwise not occur.

Drug-induced hepatitis is often caused by the formation of reactive metabolites, which may lead to either toxic hepatitis or immune system-mediated liver toxicity [37]. Unlike the related antiandrogen nilutamide, FLU was not noticeably reduced to a nitroanion free radical by NADPH-cytochrome P450 reductase. Instead, rat and human microsomal cytochrome P450 oxidatively metabolized FLU to electrophilic metabolite(s), which bound covalently to microsomal proteins [3]. However, the production of nitroanion free radical is also possible [38]. When FLU was added to rat hepatocyte and PMN cocultures, significant increase in cytotoxicity was observed which was not observed when FLU was added to rat hepatocytes and PMNs separately. This suggests that a cytochrome P450-generated metabolite of FLU produced by hepatocytes is a more potent stimulus for activation of PMNs than FLU itself [9]. Further studies are required to confirm that FLU and/or its metabolite(s) are responsible for FLU-induced hepatotoxicity with or without inflammation.

FLU may also target hepatic mitochondria and may exert oxidative stress that can lead to overt hepatic injury [39]. In the current study, decreased % MMP with/without the inflammation system was found for FLU indicating its potential as a mitochondrial toxin (Table 1). FLU (50 *µ*M) markedly inhibited respiration (mainly at the level of complex I) in isolated male rat liver mitochondria and at higher concentrations (1 mM) decreased ATP levels in isolated male rat hepatocytes [6].

A significant decrease in GSH levels (Figure 5) was also observed when FLU was administered with the H_2_O_2_ generating system and peroxidase to isolated rat hepatocytes, potentially increasing hepatocyte susceptibility to oxidant-mediated injury. This was prevented by 1 mM NAC (Figure 5). NAC is frequently used as an acetylated precursor for GSH in hepatocytes. The usefulness of NAC in modulating different diseases that include cardiovascular diseases, cancer, and chemical/metal toxicity has been reviewed by Zafarullah and colleagues [40]. Previous studies reported that FLU decreased the GSH/GSSG ratio and total protein thiols. This was associated with an early increase in phosphorylase a activity (a Ca^2+^ dependent enzyme) and a decrease in cytoskeleton-associated protein thiols, the formation of plasma membrane blebs, the release of LDH, and a loss of cell viability [3, 6]. The addition of cystine (a GSH precursor) increased GSH and decreased LDH release in male rat hepatocytes [6]. A novel GSH conjugate of FLU was reported in human liver microsomes, suggesting that the P450-mediated oxidation of FLU via a nitrogen-centered free radical could be one of several bioactivation pathways of FLU [41].

Antioxidants such as Trolox (1 mM), resveratrol (50 *µ*M), and DPPD (2 *µ*M) significantly decreased FLU + H_2_O_2_ generating system + HRP system-induced cytotoxicity and LPO and increased % MMP (Table 1) and GSH levels (Figure 5) compared to control hepatocytes. Trolox is a hydrophilic analogue of vitamin E and an established intracellular free radical scavenger [42]. Resveratrol is both a free radical scavenger and a potent antioxidant because of its ability to promote the activities of a variety of antioxidant enzymes [43]. It has three different antioxidant mechanisms: (i) competition with coenzyme Q to decrease the oxidative chain complex, the site of ROS generation, (ii) scavenging of O_2_^•−^ radicals formed in the mitochondria, and (iii) inhibition of LPO induced by the Fenton reaction products [44]. DPPD has been reported to enlarge the pool size of lipid soluble antioxidants in the whole liver cells, especially in the cytoplasmic membranes. It has also been reported to decrease LPO [45]. A significant protection against FLU-induced cytotoxicity with the H_2_O_2_ generating system and peroxidase was also achieved by a ROS scavenger, TEMPOL (200 *µ*M). TEMPOL and other stable nitroxide radicals have long been known to protect from a variety of oxidative stress-mediated injuries in laboratory animals. It can mimic superoxide dismutase activity. It can also inhibit Fenton chemistry by the ability to oxidize transition metal ions, terminate radical chain reactions by radical recombination, and accept electrons from mitochondrial electron transport chains [46]. TEMPOL was also reported to inhibit MPO-mediated protein nitration [47].

## 5. Conclusions

This study suggests that FLU-induced cytotoxicity may be increased by FLU- (or its metabolites) generated prooxidant radicals and other ROS leading to GSH depletion, increased LPO, and mitochondrial toxicity. These results raise the possibility that the presence or absence of inflammation may be another susceptibility factor for drug-induced hepatotoxicity. Using the* in vitro* oxidative stress inflammation system, it is partly possible to mimic the products formed by the inflammatory immune cells and study the mechanism of inflammation-enhanced drug-induced cytotoxicity.

## Figures and Tables

**Figure 1:** Chemical structure of flutamide.

**Scheme 1:** Simplified schematic representation of the hypothesis and aims of the study.

**Figure 2:** Respiratory burst initiated by NADPH oxidase (adapted from [14]).

**Figure 3:** Concentration-response curve of FLU (50–100 *µ*M) towards isolated rat hepatocytes to determine ACMS LC_50_.  ^*^Significant compared to control hepatocytes.

**Figure 4:** Effects of nontoxic H_2_O_2_ and peroxidase or Fe(II)-mediated Fenton model on FLU-induced cytotoxicity. Data are presented as mean ± SEM (*n* = 3). Refer to the Materials and Methods section for the description of the experiments performed and experimental conditions. HRP: horseradish peroxidase; G: glucose; GO: glucose oxidase; PTU: 6-*N*-propyl-2-thiouracil. ^a^Significant compared to control hepatocytes; ^b^significant compared to 75 *µ*M FLU; ^c^significant compared to 75 *µ*M FLU + G + GO + HRP; ^d^significant compared to 75 *µ*M FLU + G + GO + Fe(II)-mediated Fenton model.

**Figure 5:** FLU-induced GSH depletion (measured at 30 min). Refer to the Materials and Methods section for the description of the experiments performed and experimental conditions. GSH: reduced glutathione; G: glucose; GO: glucose oxidase; HRP: horseradish peroxidase; PTU: 6-*N*-propyl-2-thiouracil; NAC:* N*-acetylcysteine; Trolox: (±)-6-hydroxy-2,5,7,8-tetramethylchroman-2-carboxylic acid; resveratrol: 3,5,4′-trihydroxy-*trans*-stilbene; TEMPOL: 4-hydroxy-2,2,6,6-tetramethylpiperidin-1-oxyl; DPPD:* N,N*′-diphenyl-*p*-phenylenediamine.  ^*^Significant compared to control (only hepatocytes). ^#^Significant compared to 75 *µ*M FLU.  ^¶^Significant compared to 75 *µ*M FLU + H_2_O_2_ generating system + PTU.

**Table 1:** FLU-induced cytotoxicity and oxidative stress using an *in vitro* oxidative stress inflammation system in isolated rat hepatocytes.

Addition	Cytotoxicity (trypan blue uptake, %)			LPO (MDA, *µ*M)	MMP (% control)
Incubation time	60 min	120 min	180 min	30 min	30 min

Control	19 ± 1	21 ± 1	24 ± 1	0.30 ± 0.01	100
+H_2_O_2_ generating system + HRP	21 ± 1	23 ± 1	26 ± 1	0.33 ± 0.01	97 ± 1
+75 *µ*M FLU	30 ± 2^a^	53 ± 1^a^	66 ± 1^a^	0.48 ± 0.02^a^	86 ± 1^a,b^
+H_2_O_2_ generating system + HRP	53 ± 2^a,b^	72 ± 2^a,b^	88 ± 2^a,b^	0.60 ± 0.01^a,b^	72 ± 1^a,b^
+5 *µ*M PTU	41 ± 2^a,b,c^	56 ± 1^a,c^	72 ± 1^a,b,c^	0.53 ± 0.01^a,b^	85 ± 1^a,c^
+1 mM NAC	33 ± 2^a,c^	53 ± 1^a,c^	62 ± 1^a,c^	0.53 ± 0.02^a,b^	90 ± 1^a,b,c^
+1 mM Trolox	30 ± 1^a,c^	47 ± 1^a,c^	53 ± 1^a,b,c^	0.43 ± 0.02^a,c^	93 ± 1^a,b,c^
+50 *μ*M resveratrol	31 ± 1^a,c^	50 ± 1^a,c^	62 ± 1^a,c^	0.40 ± 0.02^a,c^	90 ± 1^a,b,c^
+200 *μ*M TEMPOL	31 ± 1^a,c^	52 ± 2^a,c^	57 ± 2^a,b,c^	0.40 ± 0.01^a,c^	88 ± 1^a,b,c^
+2 *µ*M DPPD	29 ± 2^a,c^	53 ± 1^a,c^	61 ± 1^a,b,c^	0.35 ± 0.01^c^	89 ± 1^a,c^

Data are presented as mean ± SEM (*n* = 3).

Refer to the Materials and Methods section for a description of the experiments performed and experimental conditions. LPO: lipid peroxidation; MMP: mitochondrial membrane potential; HRP: horseradish peroxidase; PTU: 6-*N*-propyl-2-thiouracil; NAC: *N*-acetylcysteine; Trolox: (±)-6-hydroxy-2,5,7,8-tetramethylchroman-2-carboxylic acid; resveratrol: 3,5,4′-trihydroxy-*trans*-stilbene; TEMPOL: 4-hydroxy-2,2,6,6-tetramethylpiperidin-1-oxyl; DPPD: *N,N*′-diphenyl-*p*-phenylenediamine.

^a^Significant compared to control (only hepatocytes).

^b^Significant compared to 75 *µ*M FLU.

^c^Significant compared to 75 *µ*M FLU + H_2_O_2_ generating system + HRP.
